# Metformin exerts anticancer effects through the inhibition of the Sonic hedgehog signaling pathway in breast cancer

**DOI:** 10.3892/ijmm.2015.2217

**Published:** 2015-05-21

**Authors:** CONG FAN, YUNSHAN WANG, ZIMING LIU, YING SUN, XIUWEN WANG, GUANGWEI WEI, JUNMIN WEI

**Affiliations:** 1 Department of Chemotherapy, Cancer Center, Qilu Hospital, Shandong University, Jinan, Shandong 250012, P.R. China; 2 Department of Human Anatomy and Key Laboratory of Experimental Teratology, Ministry of Education, Shandong University School of Medicine, Jinan, Shandong 250012, P.R. China; 3 International Biotechnology R&D Center, Shandong University School of Ocean, Weihai, Shandong 264209, P.R. China; 4 Department of Emergency Medicine, The Fifth People’s Hospital, Jinan, Shandong 250022, P.R. China

**Keywords:** metformin, Sonic hedgehog signaling pathway, cancer stem cells, AMP-activated protein kinase, breast cancer

## Abstract

Metformin, a widely prescribed antidiabetic drug, has previously been shown to lower the risk of certain types of cancer, including that of breast cancer, and to improve prognosis. Its anticancer effects, which are mediated by the activation of AMP-activated protein kinase (AMPK), have become notable. The Sonic hedgehog (Shh) signaling pathway is involved in changes in mammary ducts and malignant transformation. The aim of the present study was to elucidate the role of the Shh pathway in mediating the anticancer effects of metformin and the correlation between AMPK and the Shh pathway. We investigated the effectiveness of metformin in inhibiting the proliferation, migration, invasion and stemness of breast cancer cells *in vitro* using RNA extraction and reverse transcription-polymerase chain reaction (RT-PCR), western blot analysis, cell proliferation assay, scratch-wound assay (cell migration assay), cell invasion assay, mammosphere culture and flow cytometry. In *in vivo* experiments, a tumor xenograft model was used to detect the effects of metformin on cancer cell proliferation. The results revealed that the treatment of breast cancer cells with metformin led to the inhibition of the Shh signaling pathway. Importantly, metformin inhibited recombinant human Shh (rhShh)-induced cell migration, invasion, and stemness, and impaired cell proliferation both *in vitro* and *in vivo*. Furthermore, the small interfering RNA (siRNA)-mediated downregulation of AMPK reversed the inhibitory effects of metformin on rhShh-induced Gli-1 expression and stemness. Our findings identified a role of the Shh signaling pathway in the anticancer effects of metformin in breast cancer. Furthermore, we revealed that the metformin-mediated inhibition of the Shh signaling pathway may be dependent on AMPK.

## Introduction

Metformin is an oral biguanide agent widely used for the treatment of type 2 diabetes mellitus (1). Several studies have indicated that metformin lowers the risk of developing several types of cancer, including those of the breast, the colon and the prostate (2–5). Furthermore, metformin has been shown to inhibit cancer cell proliferation and tumor growth in animal models (6–8). The mechanisms underlying the anticancer effects of metformin vary (8,9); among these, the activation of AMP-activated protein kinase (AMPK) is pivotal (9,10). AMPK is composed of a catalytic subunit (α1 or α2) and 2 regulatory subunits (β1 or β2 and γ1, γ2 or γ3) (11). Previous studies have confirmed that the activation of AMPK by metformin is involved in mediating the anticancer effects of metformin, with metformin-induced AMPK activation leading to the inhibition of mTOR and a reduction in global translation initiation (12,13).

The Sonic hedgehog (Shh) signaling pathway is critical to cell growth and differentiation during embryonic development (14). The Shh signaling cascade is initiated when the Shh ligand binds to the cell surface receptor Patched (Ptc), which then releases its inhibitory hold on Smo. Subsequently, Smo attains the ability to transduce the signal by activating the transcriptional activator form of Gli-1, which regulates the expression of target genes that control cell growth, survival and differentiation in various types of tissue (15–17). Previous studies have demonstrated the ligand-dependent constitutive activation of the Shh pathway in several types of tumors, including those of the breast (18,19). Another study further demonstrated that a high mRNA expression of Shh, Ptc, Gli-1 and Smo in breast cancer tissue correlates with breast cancer cell invasiveness (20). Therefore, targeting the aberrant activation of the Shh signaling pathway may represent a novel treatment regime for breast cancer. Moreover, metformin has been found to have an effect on the Shh signaling pathway. A recent study indicated that metformin suppresses Shh expression in pancreatic cancer cells (21). However, it only showed that metformin reduced the expression of Shh in the BxPC3 pancreatic cancer cell line. It still remains unclear as to whether metformin exerts anticancer effects through the Shh pathway.

Breast cancer is derived from and maintained by a fraction of self-renewing tumor-initiating cells, referred to as cancer stem cells (CSCs) (22–24). Similar to other stem cells, CSCs possess the ability of self-renewal and can differentiate into various types of cancer cells (25,26). Pervious studies have identified pivotal roles for CSCs in tumor growth, invasion, metastasis and resistance to chemotherapy (27,28). A human breast cancer cell population characterized by a CD44^+^/CD24^−^ surface marker profile has been reported to be highly enriched in CSCs (25,29). However, the molecular mechanisms regulating the maintenance, self-renewal and differentiation of breast CSCs (BCSCs) remain poorly understood.

While an increasing number of studies have demonstrated the antitumor effects of metformin, little is known regarding the underlying mechanisms through which metformin affects breast cancer development. In particular, the role of the Shh signaling pathway in the anticancer effects of metformin in breast cancer remains unclear. In the present study, we initially investigated whether metformin decreases neoplastic cell proliferation and selectively kills CSCs through the Shh signaling pathway in human breast cancer. We also explored the possible association between the Shh signaling pathway and AMPK.

## Materials and methods

### Cell culture

The MDA-MB-231, MCF-7 and BT-549 human breast cancer cell lines were obtained from the American Type Culture Collection (ATCC; Manassas, VA, USA). The MDA-MB-231 and BT-549 cells were cultured in RPMI-1640 medium (Invitrogen, Carlsbad, CA, USA) supplemented with 10% fetal bovine serum (FBS; Gibco, Carlsbad, CA, USA) and 1% penicillin/streptomycin. The MCF-7 cells were grown in Dulbecco’s modified Eagle’s medium (DMEM; Invitrogen, Carlsbad, CA, USA) supplemented with 10% FBS and 1% penicillin/streptomycin. The cells were maintained at 37°C in a humidified atmosphere with 5% CO_2_.

### RNA interference

Small interfering RNA (siRNA) specific to AMPKα1 was synthesized by Shanghai GeneChem Co., Ltd. (Shanghai, China) with the following target sequences: PRKAA1-RNAi-24250-1 (siAMPK#1), TAAAGTAGCTGTGAAGATA; PRKAA1-RNAi-24251-1 (siAMPK#2), ATGCAAAGATAGCTGATTT; PRKAA1-RNAi-24252-1 (siAMPK#3), GGTCCATAGAGATTTGAAA; control siRNA (siAMPK Ctr), TTCTCCGAACGTGTCACGT. The cells were seeded in dishes until they grew to 80% confluence, and at the appointed time they were transfected with AMPKα1 siRNA or siCtr using Lipofectamine 2000 transfection reagent (Invitrogen) according to the manufacturer’s instructions. The AMPKα1 siRNA that effectively inhibited the expression of AMPK at the protein level was used in the following experiments. MDA-MB-231 cells not transfected with AMPKα1 siRNA or siCtr were used as negative controls.

### RNA extraction and reverse transcription-polymerase chain reaction (RT-PCR)

Total cellular RNA was extracted from the untreated (controls) and metformin-treated (metformin was obtained from Sigma Chemical, St. Louis, MO, USA) breast cancer cells using TRIzol reagent according to the manufacturer’s instructions (Invitrogen). The RNA was reverse-transcribed with SuperScript II Reverse Transcriptase (Invitrogen) in the presence of oligo-dT and random primers. PCR amplifications of Shh cDNA generated a product of 477 bp using the forward primer, 5′-CGCACGGGGACAGCTCGGAAGT-3′ and the reverse primer, 5′-CTGCGCGGCCCTCGTAGTGC-3′. The product of Smo was 322 bp with the forward primer, 5′-TTACCTTCAGCTGCCACTTCTACG-3′ and the reverse primer, 5′-GCCTTGGCAATCATCTTGCTCTTC-3′. The product of Ptc was 215 bp with the forward primer, 5′-TCTGCAGCAACTATACGAGC-3′ and the reverse primer, 5′-GAACAGCTCGACCGTCATCA-3′. The product of Gli-1 was 363 bp with the forward primer, 5′-GGACAACCGCCATCC AGACT-3′ and the reverse primer, 5′-GCCAGGGACACCTCCATCTC-3′. The product of GAPDH was 697 bp with the forward primer, 5′-TCACCATCTTCCCAGGAGCGAG-3′ and the reverse primer, 5′-TGTCGCTGTTGAAGTCAGAG-3′. The PCR products were analyzed by DNA gel electrophoresis on a 1% agarose gel and the intensity of each band was quantified using BandScan software. The relative expression levels of Shh, Smo, Ptc and Gli-1 were normalized to the intensity of the GAPDH bands, which served as a loading control; data are presented as the means ± standard deviation (SD).

### Western blot analysis

Cells in a monolayer culture were washed 3 times with ice-cold PBS and lysed in RIPA buffer containing protease inhibitor cocktail (Roche Diagnostics Corp., Indianapolis, IN, USA). The cell debris was removed by centrifugation at 14,000 × g for 20 min at 4°C. Protein concentrations were determined using an enhanced BCA protein assay kit (Beyotime Institute of Biotechnology, Jiangsu, China). The lysates were dissolved in Laemmli buffer, boiled for 5 min and separated (20–30 *µ*g protein per lane) by SDS-PAGE (10%), followed by electrotransfer onto polyvinylidene difluoride membranes. After blocking in 5% bovine serum albumin (BSA) in Tris-buffered saline containing Tween-20 (TBST) for 2 h at room temperature, the membranes were incubated with primary antibody at 4°C overnight. Subsequently, the membranes were washed with TBST 3 times followed by incubation with peroxidase-conjugated secondary anti-mouse (sc-390944) or anti-rabbit (sc-292373) antibodies (1:10,000; Santa Cruz Biotechnology, Inc., Santa Cruz, CA, USA) at room temperature for 1 h. After washing again with TBST 3 times, proteins were detected using the ECL Western blotting detection kit (Bio-Rad Laboratories, Hercules, CA, USA). The primary antibodies employed included anti-β-actin (1:2,000; Cat. no. 3700s; Cell Signaling Technology, Danvers, MA, USA), anti-Smo (1:1,000; ab-38686; Cell Signaling Technology), anti-Gli-1 (1:1,000; Cat. no. 3538s; Cell Signaling Technology), anti-Ptc (1:1,000; Cat. no. 2468s; Cell Signaling Technology), anti-AMPK (1:1,000; Cat. no. 2795s; Cell Signaling Technology) and anti-Shh (1:1,000; Cat. no. sc-9024; Santa Cruz Biotechnology, Inc.) antibodies.

### Cell proliferation assay

The cells were seeded in 96-well plates in complete culture medium, and after 24 h of growth, the cells were exposed to recombinant human Shh (rhShh) (1 *µ*g/ml; R&D Systems, Minneapolis, MN, USA), metformin (3 mM) or a combination of both. Following further incubation at 37°C in a humidified atmosphere with 5% CO_2_, 50 *µ*l of 3-(4,5-dimethylthiazol-2-yl)-2,5-diphenyltetrazolium bromide (MTT) stock solution (5 mg/ml; Sigma Chemical) were added to each well at the 0, 12, 24, 48 or 72 h time points, and the plates were incubated for an additional 4 h at 37°C. The solution was then removed from each well, and 150 *µ*l of dimethyl sulfoxide were added. Following gentle agitation, the absorbance at 490 nm was measured using an EL800 microplate reader (Bio-Tek Instruments, Winooski, VT, USA). Experiments were independently performed in triplicate, and 4 parallel samples were measured each time.

### Colony formation assay

The MCF-7 and MDA-MB-231 cells were trypsinized, and 500 viable cells were subcultured in 60-mm plates containing complete medium. Each treatment condition was conducted in triplicate. After 3 weeks of growth, the cells were fixed and stained with a solution containing 0.5% crystal violet and 25% methanol in water. After staining, the cells were washed with PBS. Visible colonies were macroscopically counted according to the cell numbers in each colony. All experiments were repeated 3 times.

### Tumor xenografts in BALB/c-nu mice

Six-week-old female BALB/c-nu mice were obtained from the Shanghai Slac Laboratory Animal Co., Ltd. (Shanghai,China). The mice were maintained in a specific pathogen-free facility. All experimental protocols were reviewed by the Committee on the Ethics of Animal Experiments of Shandong University (Jinan, China) and were carried out according to the Guidelines for Animal Experiments of Shandong University. MDA-MB-231 cells (1.0×10^6^) expressing green fluorescent protein (GFP) were injected subcutaneously into the abdominal mammary fat pads of these mice after they had become accommodated to their new environment. The mice had continuous free access to sterilized food and autoclaved water. When the tumor size was approximately 4 mm in diameter, the animals were randomly divided into 4 groups (3 mice per group), and treatment was initiated via intratumoral injections of rhShh alone (1 mg/kg body weight, once daily for 28 days;), oral gavage of metformin alone (100 mg/kg body weight, once daily for 28 days), as previously described (30), or a combination of both drugs. Tumor growth was compared with that of the controls (untreated mice). The mice were observed daily for any discomfort and were weighed every third day in order to detect tumor growth.

### Detection of bioluminescence

The mice were anesthetized with a 2% isoflurane/air mixture and were administered a single intraperitoneal dose of 150 mg/kg D-luciferin (Promega, Madison, WI, USA) in PBS. Images were acquired between 5 and 15 min following the administration of luciferin, and the peak luminescence signal was recorded using the *in vivo* bioluminescence imaging system (IVIS) (IVIS Spectrum; Xenogen, Hopkinton, MA, USA). The Living Image software package was used to measure photon flux within a region of interest to quantify the bioluminescence imaging signals emanating from the tumors.

### Immunohistochemical analysis

Following bioluminescence imaging, the mice were sacrificed by exposure to 1-3% isoflurane and the tumor tissues were excised, fixed and serially sectioned. Tumors derived from the transplanted cells were fixed in 10% buffered neutralized formalin for 48 h and embedded in paraffin. Consecutive sections (4-*µ*m-thick) were cut and processed for immunohistochemistry with anti-Gli-1 antibodies (1:100 dilution). Briefly, the tissue sections were deparaffinized with xylene, dehydrated with a graded series of alcohols and then incubated in 3% (v/v) hydrogen peroxide for 10 min at room temperature. Following 3 washes of 3 min each in PBS, the tissue sections were microwaved for 20 min in 10 mM citrate buffer (pH 6.0). Subsequently, the sections were washed a further 3 times in PBS for 5 min each, and incubated with normal goat serum to reduce non-specific binding. The tissue sections were then incubated with rabbit polyclonal anti-Gli-1 antibodies (1:100 dilution) at 4°C overnight. The sections were washed 3 times in PBS and biotinylated goat anti-mouse serum IgG (SP-9000; Beijing Zhongshan Golden Bridge Biotechnology, Beijing, China) was used as a secondary antibody. After washing 3 times in PBS, the sections were incubated in streptavidinbiotin conjugated with horseradish peroxidase, and the peroxidase reaction was developed with 3,3′-diaminobenzidine tetrahydro-chloride. Nuclei were counterstained with hematoxylin. The slides were examined under a light microscope, and representative images were captured from a minimum of 5 different slides from each group. Gli-1 immunostaining was regarded as positive with brown granules exhibited in the cytoplasm of a cell.

### Scratch-wound assay for the measurement of cell migration

The cells were plated in 60-mm culture dishes, and wounds were inflicted upon the cell monolayers using a sterile plastic 200-*µ*l micropipette tip. Phase-contrast microscopy images were obtained immediately after wounding and again 48 h later. The experiments were independently performed in triplicate, and the migration distance under each condition was assessed by analyzing the images using Adobe Photoshop (Adobe Systems, San Jose, CA, USA).

### Cell invasion assay

BD Matrigel-coated (BD Biosciences, San Jose, CA, USA) Transwell inserts (6.5 mm; Corning Costar Corp., Cambridge, MA, USA) containing polycarbonate filters with 8-*µ*m pores were used in the assay. The inserts were coated with 50 *µ*l of Matrigel matrix (1 mg/ml) according to the manufacturer’s recommendations. The cells were seeded in the inserts, placed in the upper chambers at a density of 2×10^5^ cells in 200 *µ*l serum-free medium, and 600 *µ*l normal growth medium was placed in the lower chambers. Following 24 h of treatment, the cells on the upper surface of the membrane were removed, and the cells on the lower chamber were fixed in 4% paraformaldehyde and stained with 0.5% crystal violet. For each membrane, the number of migratory and invasive cells in 5 random fields was counted at ×40 magnification. The experiments were performed in triplicate.

### Mammosphere culture

The cells were trypsinized and mechanically disrupted to obtain single-cell suspensions. The single-cell suspensions were then plated in Ultra-Low attachment multi-well plates (96-well plates; Corning Costar Corp.) at different densities of viable cells in serum-free mammary epithelial growth medium supplemented with 1:50 B27 (Invitrogen), 20 ng/ml epithelial growth factor, 20 ng/ml basic fibroblast growth factor (BD Biosciences) and 10 *µ*g/ml heparin (Sigma) for 7-10 days. The mammospheres were imaged and counted under a phase-contrast microscope (IX70; Olympus, Tokyo, Japan).

### Flow cytometric analysis of CD44 and CD24 expression

Cells growing in 60-mm dishes were washed once with PBS and then harvested with 0.05% trypsin/0.025% EDTA. The cell suspensions were washed with PBS and resuspended in wash buffer (1% BSA in PBS). The cells (106/100 *µ*l) were then incubated with combinations of fluorochrome-conjugated monoclonal antibodies against human CD44-APC (Cat. no. 559942; BD Biosciences), CD24-PE (Cat. no. 555428; BD Biosciences) or IgG isotype controls for APC and PE (BD Biosciences) in the dark for 30 min on ice. The labeled cells were washed with PBS and then analyzed using a FACSCalibur flow cytometer (BD Biosciences).

### Statistical analysis

Data are presented as the means ± SD with experiment numbers indicated in the figure legends. Differences between means were assessed using the Student’s two-tailed t-test. The level of significance was set at P<0.05. Statistical analysis was performed using SPSS/Win11.0 software (SPSS, Inc., Chicago, IL, USA).

## Results

### Metformin decreases Shh, Smo, Ptc and Gli-1 expression in breast cancer cells

To determine whether metformin inhibits the Shh signaling pathway in breast cancer cells, RT-PCR was employed to measure the Shh, Smo, Ptc and Gli-1 mRNA levels following treatment with metformin. The MDA-MB-231 cells were treated with various concentrations of metformin (0–9 mmol/l), as previously described (31), for 12 h or with 3 mM metformin for different periods of time (0–12 h). As shown in Fig. 1A and E, the mRNA expression levels of Shh, Smo, Ptc and Gli-1 decreased in a dose- and time-dependent manner following treatment with metformin. The changes in Shh, Smo, Ptc and Gli-1 protein expression observed in these cells following incubation with various concentrations of metformin for 12 h or with 3 mM metformin for different periods of time (0–12 h) were then determined by western blot analysis. Metformin also decreased the protein levels in a dose- and time-dependent manner (Fig. 1C and G). Treatment with metformin also suppressed Shh, Smo, Ptc and Gli-1 protein expression in the MCF-7 and BT-549 cells, as shown in Fig. 2.

### Metformin inhibits the rhShh-induced proliferation of breast cancer cells

To determine whether the suppression of Shh signaling by metformin contributes to the anticancer effects of the latter, we treated the cells with rhShh, a specific activator of the Shh signaling pathway. The effect of rhShh, metformin and rhShh combined with metformin on the proliferation of MCF-7 and MDA-MB-231 breast cancer cells was assessed by MTT assay. Treatment with 1 *µ*g/ml of rhShh increased the proliferation of these cells in a time-dependent manner, while treatment with metformin significantly decreased the growth of MDA-MB-231 and MCF-7 cells at 48 and 72 h after treatment (P<0.01 compared to control; Fig. 3A and B). We also found that treatment with 3 mM of metformin inhibited the effect of rhShh in both the MDA-MB-231 and MCF-7 cells, with a statistically significant difference identified at 72 h (P<0.01 compared to rhShh treatment; Fig. 3A and B). The proliferative potential of the breast cancer cells under the same conditions was also assessed by a colony formation assay. Incubation with metformin resulted in a significant decrease in both the number and size of colonies compared with the control group. In agreement with the results obtained by MTT assay, treatment with 3 mM of metformin inhibited the increase in the number and size of the colonies induced by rhShh when compared to treatment with rhShh alone (Fig. 3C and D).

### Metformin inhibits rhShh-induced tumor growth in vivo

To examine the effects of metformin on rhShh-induced tumor growth *in vivo*, a total of 1.0×10^6^ MDA-MB-231 cells expressing GFP were implanted into the mammary fat pads of BALB/c-nu mice. We then used IVIS to measure tumor growth in order to improve the quality of the quantitative results. An analysis of the bioluminescence imaging data indicated that the rhShh treatment group generated significantly larger tumors than the control group. However, the administration of metformin significantly inhibited tumor growth (Fig. 4A). Furthermore, the mice in the combined treatment group presented with tumors much smaller than those of the mice in the rhShh treatment group (Fig. 4A). An approximately 2.3-fold difference in the average signal intensity was observed between the rhShh treatment group and the combination treatment group (P<0.01; Fig. 4B).

Following bioluminescence imaging, the mice were sacrificed by exposure to 1-3% isoflurane and the tumor tissues were excised, fixed and serially sectioned. The expression levels of Gli-1 in the sections were detected using immunohistochemistry. The results revealed that Gli-1 expression was higher in the rhShh treatment group, but lower in the metformin treatment group when compared with the control group (Fig. 4C). Similarly, a lower expression of Gli-1 was observed in the sections from the mice administered combination treatment than in those in the rhShh treatment group (Fig. 4C).

### Metformin suppresses rhShh-induced breast cancer cell migration and invasion

We then investigated the effects of metformin on the migration potential of the MDA-MB-231 cells using the scratch-wound assay (for cell migration). The cells were seeded in 6-well plates, grown to confluence, and scratched using a 200-*µ*l pipette tip to create a wound. The cells were then incubated for 48 h in the presence of rhShh (1 *µ*g/ml), metformin (3 mM), or a combination of both. Phase-contrast images were obtained at the 0- and 48-h time points. When compared with the control group, the rhShh-treated MDA-MB-231 cells displayed a higher rate of migration (P<0.01), and the leading edges along the scraped area had almost integrated at 48 h (Fig. 5A and B). By contrast, treatment with metformin resulted in a significant decrease in cellular migration compared with the control group, and combination treatment with rhShh and metformin led to a marked inhibition of the rhShh-induced wound gap closure (P<0.01; Fig. 5A and B). A Transwell invasion assay was also performed to analyze the effects of treatment with rhShh (1 *µ*g/ml), metformin (3 mM), or their combination on the invasive capacity of the cells. The number of rhShh-treated cells that had migrated across both the Matrigel and the insert was 3-fold higher than that of the control group, while the number of migratory metformin-treated cells was approximately 70% that of the control group (P<0.01; Fig. 5C and D). The cells administered the combined treatment showed a markedly reduced invasive capacity compared with those treated with rhShh alone (Fig. 5C and D). These results suggest that metformin impairs the effects of rhShh in promoting cell invasion.

### Metformin inhibits rhShh-induced CSC stemness

To determine whether metformin inhibits the stemness of breast cancer cells through the suppression of the Shh signaling pathway, the MDA-MB-231 cells were cultured at a very low density (1 cell/*µ*l) in 96-well plates containing serum-free medium with rhShh (1 *µ*g/ml) alone, metformin (3 mM) alone, or a combination of both for 7 days. The cells treated with rhShh produced a greater number of and larger spheres compared with control cells (Fig. 6A and B). Treatment with metformin significantly reduced the number and size of these spheres compared with the control cells, and also inhibited the rhShh-induced development of a greater number of and larger spheres (P<0.01; Fig. 6A and B).

Subsequently, the MDA-MB-231 breast cancer cells were incubated with rhShh (1 *µ*g/ml), metformin (3 mM), or a combination of both for 48 h. The population of CD44^+^/CD24^−^ cells was then measured using flow cytometry. The cells which were exposed to rhShh had a higher proportion of CD44^+^/CD24^−^ cells compared to the controls (from 3.4 to 9.0%; P<0.01; Fig. 6C and D). Treatment with metformin induced a statistically significant decrease in the CD44^+^/CD24^−^ cell population, and combination treatment led to a marked inhibition of the increase in the proportion of CD44^+^/CD24^−^ cells induced by rhShh (P<0.01; Fig. 6C and D).

### AMPK is involved in the inhibition of the Shh signaling pathway by metformin

Previous studies have found that AMPK plays a critical role in facilitating the anticancer effects of metformin (9,10). Therefore, we then investigated whether the metformin-mediated inhibition of the Shh signaling pathway is dependent on AMPK. To inhibit AMPK expression, siRNA was used. Fig. 7A shows that the 3 sequences of AMPK siRNA (siAMPK#1, siAMPK#2 and siAMPK#3) effectively depleted AMPK expression at the protein level in the transfected MDA-MB-231 cells compared with cells transfected with siCtr. The sequence siAMPK#2-transfected cells were selected to examine the role of AMPK in the metformin-mediated inhibition of the Shh signaling pathway. Western blot analysis revealed a significant increase in Gli-1 expression following the combined treatment of MDA-MB-231 cells with rhShh and metformin, and transfection with siAMPK#2 compared with the cells transfected with siCtr or in the untransfected cells (Fig. 7B).

We subsequently determined whether AMPK is involved in the metformin-mediated suppression of BCSC stemness through the Shh signaling pathway. In the presence of rhShh and metformin, the siAMPK#2-transfected cells produced a greater number of and larger spheres compared with both the siCtr-transfected cells and the untransfected cells (P<0.01; Fig. 8). In the presence of rhShh and metformin, the siAMPK#2-transfected cells exhibited a significantly greater proportion of CD44^+^/CD24^−^ stem cell-like cells compared with both the siCtr-transfected cells and untransfected cells (P<0.01; Fig. 9). These results indicate that AMPK is involved in the inhibition of the Shh pathway by metformin.

## Discussion

The findings of the present study suggest that metformin significantly inhibits the Shh signaling pathway. Most importantly, our findings, to the best of our knowledge, for the first time demonstrate that metformin exerts anticancer effects through the inhibition of the Shh signaling pathway in breast cancer. Metformin is a widely used and well-tolerated oral antidiabetic agent used in the treatment of type 2 diabetes. A previous study identified that the use of metformin in patients with type 2 diabetes was associated with a lower risk of breast cancer (32). Furthermore, metformin has been found to inhibit the growth of breast cancer (33) and selectively kill CSCs (7,34). Our findings are in agreement with those of previous studies (7,33) showing that treatment with metformin significantly inhibits the growth of breast cancer cells in both MTT and colony formation assays. We further examined the effects of metformin on tumor growth *in vivo*, and showed that the tumors exposed to metformin were significantly smaller than the relevant control tumors. Additionally, we demonstrated that treatment with metformin inhibited breast cancer cell migration and invasion as well as CSC survival and self-renewal.

Studies have demonstrated that the dysregulation of the Shh signaling pathway contributes to the formation and progression of human cancers, including breast cancer (18,35). Recently, Nakamura *et al* (21) demonstrated that metformin reduces the expression of Shh in pancreatic cancer cells, suggesting that the suppression of Shh signaling is a possible mechanism through which metformin mediates its anticancer effects. We further extended this previous research to investigate the role of the Shh signaling pathway in the anticancer effects of metformin. In our analysis, a significant dose- and time-dependent decrease in the expression levels of Shh, Smo, Ptc and Gli-1 was observed in the breast cancer cells treated with metformin. In order to examine the correlation between the anticancer effects of metformin and its inhibitory effect on the Shh signaling pathway more thoroughly, we treated the cells with rhShh (a specific activator of the Shh signaling pathway). We observed that metformin significantly impaired the rhShh-induced cell proliferation *in vitro* and *in vivo*, and inhibited the migratory and invasive capacity of the cells treated with rhShh. Metformin also suppressed the increase in the proportion of CD44^+^/CD24^−^ cells and the development of a greater number of and larger spheres induced by rhShh. These findings support a central role for the inhibition of the Shh signaling pathway in mediating the anticancer effects of metformin in breast cancer.

Based on the aforementioned findings, we further investigated whether the metformin-mediated inhibition of the Shh signaling pathway is AMPK-dependent. The activation of AMPK was identified as pivotal in enabling the anticancer effects of metformin. Following the downregulation of AMPKα1 expression by siRNA, the cells were treated with rhShh and metformin. A significant increase in Gli-1 expression was observed in the cells transfected with siRNA against AMPKα1 compared with the cells transfected with the control siRNA or the untransfected cells. The downregulation of AMPKα1 expression reversed the inhibitory effects of metformin on rhShh-induced Gli-1 expression. AMPK was also shown to be involved in the metformin-mediated suppression of BCSC stemness through the Shh signaling pathway. This suggests that the inhibition of the Shh signaling pathway mediated by metformin occurred through an AMPK-dependent mechanism.

Although further research is required to clarify the mechanisms underlying the anticancer effects of metformin, the present study demonstrates that the inhibition of the Shh signaling pathway is a significant contributing factor to the anticancer effects of metformin in breast cancer. Additionally, we identified that the metformin-mediated inhibition of the Shh signaling pathway is dependent on AMPK.

In conclusion, to the best of our knowledge, the present study is the first to identify that metformin exerts anticancer effects through the inhibition of the Shh signaling pathway in breast cancer. The downregulation of Shh signaling by metformin inhibited the proliferation of cancer cells both *in vitro* and *in vivo*, impaired cellular migration and invasion, and reduced BCSC survival and self-renewal capacity. Furthermore, the metformin-mediated inhibition of the Shh signaling pathway was partially dependent on AMPK. However, further research is required on the molecular mechanisms of the association between the anticancer effects of metformin and the Shh signaling pathway.

## Figures and Tables

**Figure 1:** Metformin decreases Sonic hedgehog (Shh), Smo, Patched (Ptc) and Gli-1 expression in MDA-MB-231 cells. MDA-MB-231 cells were treated with metformin at concentrations of 0, 1, 3 or 9 mM for 12 h or with 3 mM of metformin for 0, 3, 6 and 12 h. (A and E) The mRNA levels of Shh, Smo, Ptc and Gli-1 were measured by RT-PCR; GAPDH served as a control. (C and G) The protein levels of Shh, Smo, Ptc and Gli-1 were measured by western blot analysis; β-actin levels were measured as a loading control. Histograms illustrate the (B and F) mRNA levels relative to those of GAPDH and (D and H) protein expression relative to that of β-actin. All data are presented as the means ± SD of 3 independent experiments. ^*^P<0.05 vs. the control group; ^**^P<0.01 vs. the control group.

**Figure 2:** Metformin decreases Sonic hedgehog (Shh), Smo, Patched (Ptc) and Gli-1 expression in MCF-7 and BT-549 cells. (A and C) Western blot analysis was used to detect Shh, Smo, Ptc and Gli-1 expression in the MCF-7 and BT-549 cells. β-actin was used as a loading control. (B and D) Histograms illustrate protein expression relative to that of β-actin. All data are presented as the means ± SD of 3 independent experiments. ^**^P<0.01 vs. the control group.

**Figure 3:** Metformin inhibits the recombinant human Sonic hedgehog (rhShh)-induced proliferation of breast cancer cells. (A and B) MTT assay of MDA-MB-231 and MCF-7 cells was conducted at 0, 12, 24, 48 and 72 h. All data represent the means ± SD of 3 separate experiments performed in triplicate. ^**^P<0.01 vs. the control (Ctr) group, ^##^P<0.01 vs. the rhShh group. (C and D) Colony formation assays of MDA-MB-231 and MCF-7 cells. The number of colonies was counted under a microscope. ^**^P<0.01 vs. the Ctr group; ^##^P<0.01 vs. the rhShh group.

**Figure 4:** Metformin inhibits recombinant human Sonic hedgehog (rhShh)-induced tumor growth in the *in vivo* model of breast cancer. (A) Representative bioluminesence images of the control and the treatment groups: control (ctr; untreated), rhShh (intratumoral injections of rhShh, 1 mg/kg body weight), Met (oral gavage of metformin, 100 mg/kg body weight), Met + rhShh (a combination of both drugs). (B) Chart representing the average photon counts from the control and the treatment groups. The bars indicate the means ± SD of triplicate samples, ^**^P<0.01 vs. the Ctr group, ^##^P<0.01 vs. the rhShh group. (C) The expression levels of Gli-1 in the tumors from the xenograft model were measured by immunohistochemistry. Gli-1 immunostaining was regarded as positive with brown granules exhibited in the cytoplasm of a cell. Final magnification, ×40. Scale bar, 50 *µ*m.

**Figure 5:** Metformin suppresses the rhShh-induced cell migration and invasion. (A) Representative images of the wounds at 0 and 48 h in the presence of recombinant human Sonic hedgehog (rhShh), metformin or their combination. (B) Histogram illustrates the relative wound width at 0 and 48 h. The migration distance of each cell was measured using Adobe Photoshop. (C) Matrigel invasion assay. Cells were seeded into Matrigel-coated invasion chambers and were treated with rhShh, metformin or their combination for 24 h. Representative images of stained and invaded cells are shown. Magnification, ×10. (D) The number of invaded cells was quantified by counting the cells from 5 random fields. All data represent the means ± SD of 3 separate experiments (^**^P<0.01 vs. the Ctr group, ^##^P<0.01 vs.the rhShh group).

**Figure 6:** Metformin inhibits rhShh-induced sphere formation and reduces the number of CD44^+^/CD24^−^ MDA-MB-231 cells. (A) Representative images of MDA-MB-231 cells in the presence of recombinant human Sonic hedgehog (rhShh), metformin and their combination. (B) The number of spheres was counted under a microscope. Data represent the means ± SD of 3 separate experiments (^**^P<0.01 vs. the Ctr group, ^##^P<0.01 vs. the rhShh group) (C) Cells were treated with rhShh, metformin and their combination. After 4 days, the cells were stained with anti-CD44-APC and anti-CD24-PE antibodies, and the CD44^+^/CD24^−^ subpopulations were examined by flow cytometry. (D) Histogram illustrates the percentages of the CD44^+^/CD24^−^ subpopulations. All data represent the means ± SD of 3 separate experiments (^**^P<0.01 vs. the Ctr group, ^##^P<0.01 vs. the rhShh group).

**Figure 7:** AMP-activated protein kinase (AMPK)α1 is involved in the inhibitory effects of metformin on the expression of Gli-1. (A) MDA-MB-231 cells were transfected with siAMPK#1 (PRKAA1-RNAi-24250-1), siAMPK#2 (PRKAA1-RNAi-24251-1), siAMPK#3 (PRKAA1-RNAi-24252-1), or siCtr, and 48 h after transfection, the cells were lysed and examined by western blot analysis; β-actin was used for loading control. (B) Untransfected MDA-MB-231 cells were treated with recombinant human Sonic hedgehog (rhShh) or the combination of rhShh and metformin, and the control group was treated with PBS. MDA-MB-231 cells were transfected with siCtr or siAMPK#2 in the presence of rhShh and metformin. Gli-1 protein levels were examined by western blot analysis. β-actin levels were measured as a loading control.

**Figure 8:** AMP-activated protein kinase (AMPK)α1 is involved in the inhibitory effect of metformin on sphere formation in MDA-MB-231 cells. (A) Representative images of MDA-MB-231 cells in the presence of recombinant human Sonic hedgehog (rhShh) or the combination of rhShh and metformin, or the cells transfected with siCtr or siAMPK#2 in the presence of rhShh and metformin. The cells (1 cell/*µ*l) were cultured in 96-well plates containing 100 *µ*l serum-free medium in each well for 7 days. (B) The number of spheres was counted under a microscope. Error bars represent the means ± SD, ^**^P<0.01 vs. the Ctr group, ^##^P< 0.01 vs. the rhShh group, ^&&^P<0.01 vs. the cells transfected with siCtr in the presence of rhShh and metformin.

**Figure 9:** The metformin-induced decrease in the number/percentage of CD44^+^/CD24^−^ MDA-MB-231 cells is dependent on AMPK. (A) MDA-MB-231 cells were treated with recombinant human Sonic hedgehog (rhShh) or the combination of rhShh and metformin; the cells were treated with sterile PBS as a control and the cells were transfected with siCtr or siAMPK#2 in the presence of rhShh and metformin. The CD44^+^/CD24^−^ subpopulations were examined by flow cytometry. (B) The histogram illustrates the percentage of CD44^+^/CD24^−^ subpopulations. Error bars represent the means ± SD; ^**^P<0.01 vs. the Ctr group, ^##^P<0.01 vs. the rhShh group, ^&&^P<0.01 vs. the cells transfected with siCtr in the presence of rhShh and metformin.
